The article "Analysis of Factors Related to Adolescents' Physical Activity Behavior Based on Multichannel LSTM Model" was retracted in 2023. Reasons: unreliable results or conclusions; concerns about the data; concerns about the results or conclusions; concerns about the peer review.

# Analysis of Factors Related to Adolescents' Physical Activity Behavior Based on Multichannel LSTM Model

**DOI:** 10.1155/2022/1022421

**Published:** 2022-07-04

**Authors:** Guiling Chang, Jinfeng Liu

**Affiliations:** ^1^Xian Universitv of Finance and Economics, Xian, Shaanxi 710100, China; ^2^The Department of Physical Education, Huainan Normal University, Anhui, Huainan 232001, China

## Abstract

The health problems of teenagers are closely related to their sports behavior. In order to understand the relevant factors of teenagers' sports behavior, we use a variety of research methods to make a brief theoretical analysis of the relevant factors of teenagers' sports behavior and analyze the impact of the model on teenagers' sports behavior from different levels. The model analyzes the factors affecting youth sports behavior, reveals the relationship between these factors, puts forward corresponding intervention strategies, and uses effective means to develop youth sports practice. Therefore, based on the analysis of the relevant factors of teenagers' sports behavior, this paper puts forward the LSTM model from many aspects, which shows that our model can be very effective in analyzing the factors affecting teenagers' sports behavior.

## 1. Introduction

The obesity rate in China has doubled in the last 30 years, according to The Times, UK. The rate of obesity and overweight among adults in developing countries increased from 250 million in 1980 to 904 million in 2008, and China now has a quarter of the obese and overweight population [1]. This study analyzes the factors influencing the physical activity behavior of adolescent students to provide a theoretical reference for physical education programs aimed at improving adolescent exercise behavior and promoting adolescent health [2].

At this stage, there are various factors that influence adolescent physical activity behavior. Individual factors are the primary factors of adolescent physical exercise behavior, which are necessary for exercise behavior. Individual physiological factors determine individual exercise behavior, and psychological factors promote the development of individual motor behavior [3]. Individual physiological factors are one of the important factors influencing adolescent physical exercise behavior, and factors such as height, weight, physical health status, and body size of adolescents are common research variables in studies. For example, [4] in a study on the formation factors of exercise habits among college students, it was pointed out that the motivation to lose weight and build physical beauty could promote the change of exercise behavior among college students, and individual athletic ability influenced by congenital genetic factors could also affect the exercise behavior of individuals. [5] The amount of physical activity of adolescents was studied in terms of gender, age, height, and weight, and the influence of physiological, psychological, sociocultural, and environmental factors on the physical activity of adolescents was studied. As far as psychological factors are concerned, there is a relationship between individual achievement and individual personality. The study of [6] has pointed out that those adolescents who are adventurous and challenging may prefer competitive sports programs, where exercise provides satisfaction and pleasure, and the act of physical activity provides individuals with the opportunity to demonstrate their level of athletic ability, strengthening their self-esteem and pride. The motivation that is motivational and persistent and determines the intensity of behavior is an essential factor in motivating individuals to participate in sports.

The article "Analysis of Factors Related to Adolescents' Physical Activity Behavior Based on Multichannel LSTM Model" was retracted in 2023. Reasons: unreliable results or conclusions; concerns about the data; concerns about the results or conclusions; concerns about the peer review.

Family factors are both physical environmental factors that satisfy the conditions and environment of adolescents' exercise, and internal psychological factors that promote individual adolescents' internal motivation and increase the level of individual exercise motivation [7]. Parents' exercise awareness and exercise behavior, cultural level, and socio-economic status are important. School physical education is the main form of physical activity behavior of young students, and it is the main channel of physical activity of young people [8]. A reasonable physical education program can stimulate students' motivation to exercise, induce behavior change, satisfy students' self-actualization and sense of accomplishment, and also explain the causes of behavior change and its internal mechanism of action [9]. However, a common phenomenon in primary and secondary schools in China is that the number of physical education classes per week, the number of recesses, and the participation in school sports all decrease with grade level, and school sports become the main place to train students who have neither the awareness nor the ability to exercise [10].

Physical education teachers are the implementers of physical education and the organizers of extracurricular physical activities, and the amount of physical activity in schools for young students is closely related to the physical education teachers. Issues such as the number of games and competitions organized in school, the physical culture of the school, and exercise peers are the main factors that limit students' exercise behavior [11]. The phenomenon of physical education classes being squeezed is an important factor that currently restricts the development of physical education in schools, and “exam-oriented education” has seriously skewed educational values, with many schools pursuing the promotion rate unilaterally and squeezing and diverting students' physical education classes and extracurricular physical activities at will.

The article "Analysis of Factors Related to Adolescents' Physical Activity Behavior Based on Multichannel LSTM Model" was retracted in 2023. Reasons: unreliable results or conclusions; concerns about the data; concerns about the results or conclusions; concerns about the peer review.

Social support, community exercise environment, and safety issues in the community were the main social level factors that governed youth physical activity behavior. Parental support, sibling support, school teacher support among school factors, and peer friend support were the main components of social support. Adolescents' perceived social support is closely related to their physical activity behavior and has a direct or indirect effect on self-efficacy. Researchers have compared parent-child communication, parental support, and adolescent psychological risk factors in obese and normal weight adolescents and found that parent-child communication and parental support had a significant impact on normal weight adolescents, while parental support had a more significant impact on obese adolescents. The lack of sports facilities is the main objective factor affecting individual exercise behavior. Studies on community exercise behavior found that the lack of public sports facilities in the community is the main factor affecting the physical exercise behavior of urban adolescents. The convenience of sports facilities and field equipment around the home, the good or bad exercise environment, and the development of sports activities all have an impact on the form of adolescent physical exercise behavior, the choice of sports, exercise attitude, exercise awareness, exercise behavior, effort, and persistence.

## 2. Related Work

The factors influencing adolescent children's physical activity behaviors were studied in terms of subjective beliefs of both parents, objective material conditions, and work-life environment [12]. The study showed that parents' physical activity behaviors play a major role in promoting the formation of adolescents' sports perceptions, and that parents' actual exercise behaviors and exercise perceptions can contribute to adolescent children's internal motivation to exercise [13]. The stronger the family members' beliefs about exercise, the better the family exercise climate, and the stronger the family members' motivation to exercise and the greater the likelihood of physical activity behaviors.

In terms of family socioeconomic status, [14] a study of the family cultural level was conducted to explore the effects of different cultural level levels of youth physical activity behavior, and the results showed that the effect of family cultural level on youth exercise perceptions reached significant levels. The higher the literacy level of parents, the greater the possibility of active intake of family education knowledge and the more scientific the attitude of educating their children. For the study of economic status, [15] concluded that parents' exercise commitment was positively associated with adolescents' exercise behavior, but the level of parental exercise commitment perceived by adolescents was low, and that adolescent children's exercise behavior would be better developed if the intensity of commitment was increased. Parental encouragement and support are particularly important for the physical activity behaviors of 13- to 16-year-olds, and physical activity behaviors need to be sustained based on parental material support.

The article "Analysis of Factors Related to Adolescents' Physical Activity Behavior Based on Multichannel LSTM Model" was retracted in 2023. Reasons: unreliable results or conclusions; concerns about the data; concerns about the results or conclusions; concerns about the peer review.

Safety issues and the safety of school sports equipment are key factors that limit physical activity and have a direct impact on youth physical activity behaviors. Studies by foreign scholars on safety have focused on whether relevant sports equipment meets national safety standards, whether schools regularly inspect sports equipment, the safe sports environment created by the joint efforts of schools and society, and the convenience of access to drinking water and sports rest areas during individual adolescent physical activity behaviors. The study of [16] found that low levels of community safety were strongly associated with physical activity levels and that residents of communities with lower levels of safety had higher rates of obesity and larger BMI indices.

Factor 1 mainly focused on reflecting motivation, interest in physical activity, sense of achievement in sports, enjoyable experience of sports, positive expectation of sports outcome, positive self-evaluation, and attitude toward sports knowledge. Among them, the sense of achievement in sports and interest in sports were the most highly correlated with F1, indicating that they are the more important factors in explaining the physical activity behavior of adolescents [17]. The sense of achievement in sports can lead to psychological tendencies of pleasure and success from the heart, which all stem from the individual's active participation in sports. Sports behavior formed by sports interest can make individuals gain more knowledge about sports and health, improve motor skills, and promote healthy physical and mental development, as well as produce pleasant emotional experiences. In addition, the motivation of sports is also a factor that should not be neglected, as shown in a study by the authors of [18], motivation for physical activity is positively correlated with exercise adherence, and extrinsic motivation motivates people to participate in physical activity. Attitudes toward physical education knowledge had a slightly lower correlation with factor 1, suggesting less importance in comparison to other factors. The study of [1] showed that students' perceived value and role of physical activity showed a high correlation (*r*=0.87) with adherence to physical activity in the long term, indicating that the perception of the value and role of physical education itself is an important factor influencing students' adherence to physical activity. This shows that there are some differences in the role played by the attitude factor of physical education knowledge in two different stages of physical activity behavior.

The article "Analysis of Factors Related to Adolescents' Physical Activity Behavior Based on Multichannel LSTM Model" was retracted in 2023. Reasons: unreliable results or conclusions; concerns about the data; concerns about the results or conclusions; concerns about the peer review.

Factor 2 concentrates on the individual's physical quality, health status, and the degree of importance. Among them, an individual's health status and physical fitness have a high correlation, and it can be said that an individual's physical fitness and health status are necessary prerequisites for realizing a variety of psychological factors and are the physical basis of physical exercise behavior. Therefore, physical health factors and psychological factors complement each other, physical health factors are the basis of psychological factors, and psychological factors play a role in promoting physical health [19].

## 3. Methods

A single-channel LSTM-based method for analyzing factors related to youth physical activity behavior mainly includes LSTMs use memory units to avoid gradient disappearance and gradient explosion during backpropagation, can learn long-term dependencies, and make full use of historical information. The LSTM was improved and extended, making it widely used in natural language processing, speech recognition, and other fields.

The LSTM unit is shown in Figure 1.

The updating process of the LSTM unit at time *t* is as follows:

(1) $$\begin{array}{c} \left.i_{t}=\sigma W_{i}x_{t}+U_{i}h_{t-1}+V_{i}c_{t-1}\right),\\ c_{t}=\tanh\left(W_{c}x_{t}+U_{c}h_{t-1}\right),\\ \left.f_{t}=\sigma W_{f}x_{t}+U_{f}h_{t-1}+V_{f}c_{t-1}\right),\\ c_{t}=f_{t}⊙c_{t-1}+i_{t}⊙c_{t},\\ \left.o_{t}=\sigma W_{o}x_{t}+U_{o}h_{t-1}+V_{o}c_{t}\right),\\ h_{t}=o_{t}⊙\;\tanh\left(c_{t}\right), \end{array}$$

where *x*_*i*_ is the input data of the memory unit, *σ* is the logistic sigmoid function, and the symbol ⊙ is the dot product operation between vectors. *i*_*t*_, *o*_*t*_, *f*_*t*_, *c*_*t*_ are the values of the input gate, output gate, forgetting gate, and memory cell at time *t*, respectively, *c*_*t*_ are the values of the candidate memory states of the memory cell and *h*_*t*_ are the outputs of the LSTM cell at time *t*.

The article "Analysis of Factors Related to Adolescents' Physical Activity Behavior Based on Multichannel LSTM Model" was retracted in 2023. Reasons: unreliable results or conclusions; concerns about the data; concerns about the results or conclusions; concerns about the peer review.

For the analysis of the factors associated with youth physical activity behavior, we obtain a balanced sample of the factors associated with each youth physical activity behavior and then used a single-channel LSTM as the classification method as shown in Figure 2. The input feature vectors are passed through the LSTM layer to obtain high-dimensional vectors, which can learn deeper features that can better describe the samples. The fully-connected layer is receiving all the outputs from the previous layer, weighting and summing these output vectors, and propagating the weighted outputs through the excitation function to the Dropout layer. In this experiment, the excitation function is shown in the following equation:

(2) $$\begin{array}{c} g\left(x\right)=\max\left(0,x\right), \end{array}$$

where *x* is the output vector and the ReLU function sets all values less than 0 to 0, with the ability to bootstrap moderate sparsity. The Dropout layer is shown in following equation:

(3) $$\begin{array}{c} g=h^{*}•D\left(p\right). \end{array}$$

Finally, the output of the single-channel LSTM model is used to classify the samples by the Softmax output layer.

(4) $$\begin{array}{c} {\text{label}}_{\text{pred}}=\arg\max_{i}P\left(Y=i|x,W,U,V\right), \end{array}$$

where *x* is the upper layer output vector, *i* is the label prediction, *W*, *U*, *V* are the coefficient matrices in the LSTM update method, and label_pred_ is the predicted label with the highest posterior probability.

The application of random undersampling and single-channel LSTM for the analysis of factors related to youth physical activity behavior has an obvious drawback: because undersampling only selects some samples from multiple classes and a large number of unselected samples. The method undersamples the imbalanced samples several times to obtain multiple sets of balanced samples, uses each set of balanced samples to learn an LSTM model, and uses the Merge layer to jointly learn multiple LSTMs.

The multichannel LSTM classifier framework is shown in Figure 3.

In the process of model training, we minimize,

(5) $$\begin{array}{c} J=-\sum_{i=1}^{N}\sum_{l=1}^{m}\left[1\left\{t_{i}=l\right\}\log\left(y_{l}\right)\right]+\frac{\lambda }{2N}\sum_{k=1}^{n}\left({\sum_{\varepsilon \in \omega }\left\|W_{\varepsilon }^{k}\right\|}_{F}^{2}+{\sum_{\varepsilon \in \mu }\left\|U_{\varepsilon }^{k}\right\|}_{F}^{2}+{\sum_{\varepsilon \in \nu }\left\|V_{\varepsilon }^{k}\right\|}_{F}^{2}\right). \end{array}$$

In the loss function, in addition to minimizing the negative log likelihood, the L2 regularization of *W*, *U*, *V* is added because the parameters of the Softmax function are redundant, i.e., the minima are not unique, and the addition of the regularization term can make the minima unique. The penalty factor *λ* regulates the weight of the regularization term, and the larger the value, the greater the penalty for large parameters.

The article "Analysis of Factors Related to Adolescents' Physical Activity Behavior Based on Multichannel LSTM Model" was retracted in 2023. Reasons: unreliable results or conclusions; concerns about the data; concerns about the results or conclusions; concerns about the peer review.

## 4. Experiments

The analysis of the contents of the family's lifestyle, the way of interaction with the children, the interaction with the children, the parents' sports knowledge structure, sports habits and sports awareness and behavior, the level of support from the relatives, and the family recreation side was carried out according to the different influencing factors. The reliability statistics under different influencing factors are in Table 1.

The factors with a high correlation with factor 1 include family sports atmosphere, family lifestyle, and tutoring style. It indicates that these factors exert an important influence in adolescent physical exercise behavior, and adolescent physical exercise behavior is often closely linked to the sports atmosphere of the family, and parents' sports ideology, attitude, awareness, and behavior habits towards sports all have a subtle influence on their children. The results in Table 2 show that exercisers and nonexercisers show significant differences in the dimensions of physical exercise attitudes.

Based on the above-given correlation analysis of each factor of exercise attitudes and the correlation analysis of exercise attitudes and physical behavior, the path relationships among the variables were further explored in conjunction with the theory relied on in this study. The path relationships among the variables were examined behavioral intentions on physical activity behaviors; and behavioral habits, behavioral attitudes, and sense of behavioral control on physical activity behaviors, while constructing path diagrams based on them.

Behavioral attitudes can have an impact on sport behavior only through the intermediate variable of behavioral perceptions, see Figure 4.

Specifically, the specific parameters we used are shown in Table 3.

Accuracy and geometric mean (G-mean) were used as a measure of classification effectiveness. The geometric mean is calculated as shown in the following equation:

(6) $$\begin{array}{c} G-\text{mean}=\sqrt[{n}]{\prod_{i=1}^{n}{\text{Recall}}_{i}}, \end{array}$$

where Recall_*i*_ denotes the recall of category *i*, *n* is the number of categories, and *n* is taken as 7 in this experiment.

In the experiment, we implemented the following methods to deal with the analysis of factors related to youth physical activity behavior:

1. Full training + maximum entropy (FullT + Maxent), all the remaining samples of each class are used as training samples and the maximum entropy classifier is used.
2. Random oversampling + maximum entropy (OverS + Maxent), let the maximum number of remaining samples of each class (preference class) be *n*_max_ and use the random oversampling technique to extract *n*_max_ samples from the remaining samples of each class as training samples, using the maximum entropy classifier.
3. Random undersampling + maximum entropy (UnderS + Maxent), let the number of remaining samples of the second smallest class (surprise class) be *n*_min_, and *n*_min_ samples from the remaining samples of each class are used as training samples using the random undersampling technique, and the maximum entropy classifier is used.
4. Random undersampling + single channel LSTM (UnderS + LS TM), using the sampling method in (3) to obtain the training samples, and the classifier uses a single channel LSTM.
5. Random undersampling + single-channel CNN (UnderS + CNN), using the sampling method in (3) to obtain the training samples, and the classifier uses a single-channel CNN.
6. Random undersampling + integrated learning (Ensemble-Maxent), multiple sets of training samples (5 sets for this experiment) are obtained using the sampling method in (3), and multiple base classifiers are built. Finally, integrated learning is performed by fusing the results of these base classifiers, where the base classifier is chosen as the maximum entropy classifier.
7. Random undersampling + multichannel LSTM (Multi-LSTM), using the sampling method in (5) to obtain multiple sets of training samples (5 sets in this experiment), and the classifier using a multichannel (5-channel) LSTM neural network [20–22].
8. Random undersampling + multichannel CNN (Multi-CNN), using the sampling method in (5) to obtain multiple sets of training samples (5 sets for this experiment), and a multichannel (5-channel) CNN for the classifier.

The article "Analysis of Factors Related to Adolescents' Physical Activity Behavior Based on Multichannel LSTM Model" was retracted in 2023. Reasons: unreliable results or conclusions; concerns about the data; concerns about the results or conclusions; concerns about the peer review.

Figure 5 compares the classification effects of fully trained, randomly oversampled, and randomly undersampled methods in the analysis of factors related to youth physical activity behavior. We can see that the random nonpublic classification is obviously better than the first two methods, and its advantage is particularly obvious in the average value of *g*. The main reason for this phenomenon is that in the complete training and random sampling methods, the classification algorithm is very inclined to take more samples by category, resulting in the number of samples being less than the feedback category.

The error accumulation results of this method are shown in Figure 6.

Next, we compare the classification performance of the maximum entropy and LSTM under the random undersampling method. Figure 6 shows that the classification performance of single-channel LSTM is better than that of maximum entropy, with an improvement of 1.8% and 1.2% in accuracy and G-mean, respectively. We analyze that the main reason is that the LSTM can use the historical information and can learn the long-term dependence between samples. In addition, we also implemented a convolutional neural network (CNN)-based classification method. From Figure 7, we can see that the classification performance of LSTM and CNN are comparable, with LSTM having a slight advantage in accuracy and CNN having a slightly higher G-mean.

In the problem of analyzing factors related to youth physical activity behavior, the undersampling-based integrated learning approach performs better to use all labeled samples while maintaining a balance between training samples. Next, we will compare the classification performance of the undersampling-based integrated learning approach with our proposed multichannel LSTM classification approach, as shown in Figure 8.

The results in Figure 8 show that the multichannel LSTM-based classification method improves 1.5% in accuracy and 2.8% in G-mean over the integrated learning method when the hidden layer features are fused using sum; the multichannel LSTM-based classification method improves 1.5% in accuracy and 2.8% in G-mean over the integrated learning method when the hidden layer features are fused using concatenate.

As in Figure 9, when the hidden features are fused using concatenate, the multichannel LSTM-based classification method improves by 1.0% in accuracy and 2.1% in G-mean over the integrated learning method. These results indicate that the multichannel LSTM-based classification method is very effective for analyzing factors related to youth physical activity behavior.

## 5. Conclusion

Factors affecting adolescents' physical activity behavior, namely, there are internal factors of individuals as well as family, school, and social factors closely related to individuals. Family sports environment and atmosphere as well as parents' sports awareness directly influence adolescents' physical activity behavior, and reliable and effective educational measures should be provided for the new generation of young parents to strengthen parents' or guardians' educational interventions on the importance of regular physical activity for adolescents in response to our special national conditions. We propose a multichannel LSTM-based analysis of factors related to adolescents' physical activity behavior, and our method is found to be very effective in the analysis of related factors. It is hoped that the subsequent trinity of school, family, and society under the guidance of relevant policies will certainly promote the physical fitness of adolescents and improve their health behaviors.

The article "Analysis of Factors Related to Adolescents' Physical Activity Behavior Based on Multichannel LSTM Model" was retracted in 2023. Reasons: unreliable results or conclusions; concerns about the data; concerns about the results or conclusions; concerns about the peer review.

## Figures and Tables

**Figure 1:** LSTM unit.

**Figure 2:** Single-channel LSTM classifier framework.

**Figure 3:** Multichannel LSTM classifier framework.

**Figure 4:** Path diagram of the influence of exercise attitude on physical behavior.

**Figure 5:** Comparison of classification performance of traditional methods for analyzing factors related to youth physical activity behavior.

**Figure 6:** Error accumulation results.

**Figure 7:** Comparison of classification performance of maximum entropy and neural networks.

**Figure 8:** Comparison of classification performance between integrated learning and multichannel neural networks.

**Figure 9:** The importance of different factors.

**Table 1:** Reliability statistics for each subscale of the influencing factors of youth physical activity behavior.

Scale level	Cronbach*α* coefficient	Standardized *α* coefficient	# Subscale question items
Individual level	0.878	0.879	12
Family level	0.915	0.916	11
School level	0.902	0.903	9
Community level	0.918	0.919	13
Policy level	0.939	0.939	10

**Table 2:** Summary of the scores of adolescents' attitudes toward physical exercise.

	Exercisers (*N* = 100)		Nonexercisers (*N* = 251)		T	*P*
	M	SD	M	SD		
Behavioral attitudes	31.0500	4.759	26.4548	4.915	7.968	0.0001
Target attitudes	48.6500	8.042	45.7812	6.051	3.678	0.0001
Behavioral cognition	29.0600	3.555	27.9525	3.309	0.878	0.004
Behavioral habits	37.1500	6.305	31.1995	6.405	7.885	0.0001
Behavioral intention	27.3200	3.502	24.1875	4.018	6.815	0.0001
Emotional experience	38.1800	5.855	34.2235	5.845	5.715	0.0001
Behavioral control	25.1500	4.935	20.9845	4.161	7.989	0.0001
Subjective standards	18.3800	4.295	20.7575	3.999	−4.865	0.0001

**Table 3:** Parameter settings in the LSTM.

Parameter expression	Parameter value
Input vector length	120
LSTM layer output dimension	128
Fully connected layer output dimension	64
Dropout parameter	0.5
#iterations	20

## Data Availability

The experimental data used to support the findings of this study are available from the corresponding author upon request.
